The article "microRNA‐374 inhibits proliferation and promotes apoptosis of mouse melanoma cells by inactivating the Wnt signalling pathway through its effect on tyrosinase" was retracted in 2021. Reasons: errors in the images; unreliable results or conclusions.

# microRNA‐374 inhibits proliferation and promotes apoptosis of mouse melanoma cells by inactivating the Wnt signalling pathway through its effect on tyrosinase

**DOI:** 10.1111/jcmm.14348

**Published:** 2019-06-17

**Authors:** Xiao‐Jing Li, Zhi‐Feng Li, Yan‐Yan Xu, Zhao Han, Zhi‐Jun Liu

**Affiliations:** ^1^ Department of Dermatology Affiliated Hospital of Hebei Engineering University Handan P. R. China

**Keywords:** apoptosis, melanoma, microRNA‐374, proliferation, TYR gene, Wnt signalling pathway

## Abstract

Melanoma is one of the most malignant skin tumours with constantly increasing incidence worldwide. Previous studies have demonstrated that microRNA‐374 (miR‐374) is a novel biomarker for cancer therapy. Therefore, this study explores whether miR‐374 targeting tyrosinase (TYR) affects melanoma and its underlying mechanism. We constructed subcutaneous melanoma models to carry out the following experiments. The cells were transfected with a series of miR‐374 mimics, miR‐374 inhibitors or siRNA against TYR. Dual luciferase reporter gene assay was used for the verification of the targeting relationship between miR‐374 and TYR. Reverse transcription quantitative polymerase chain reaction and western blot analysis were conducted to determine the expression of miR‐374, TYR, β‐catenin, B‐cell leukaemia 2 (Bcl‐2), Bcl‐2 associated X protein (Bax), Low‐density lipoprotein receptor‐related protein 6 (LRP6), Leucine‐rich repeat G protein‐coupled receptor 5 (LGR5) and CyclinD1. Cell proliferation, migration, invasion, cell cycle distribution and apoptosis were evaluated using cell counting kit‐8 assay, scratch test, transwell assay and flow cytometry respectively. TYR was proved as a putative target of miR‐374 as the evidenced by the result. It was observed that up‐regulated miR‐374 or down‐regulated TYR increased expression of Bax and decreased expressions of TYR, β‐catenin, LRP6, Bcl‐2, CyclinD1 and LGR5, along with diminished cell proliferation, migration, invasion and enhanced apoptosis. Meanwhile, cells with miR‐374 inhibitors showed an opposite trend. These findings indicated that up‐regulated miR‐374 could inhibit the expression of TYR to suppress cell proliferation, migration, invasion and promote cell apoptosis in melanoma cells by inhibiting the Wnt signalling pathway.

## 1 INTRODUCTION

Melanomas are one of the malignant neoplasms of melanocytes, which develop mainly in the skin, although they can be occasionally develop in the central nervous system, mucous membranes and eyes.^1^ Melanomas are a type of common immunogenic tumours in many neoplasms that are often non‐responsive to immunotherapy.^2^ Malignant forms of melanomas are most commonly derived from the neural crest lineage and spread quickly from the localized cutaneous disease to the regional lymph node, which could result in more advanced visceral metastasis.^3^ Although melanoma is a relatively rare form of cancer, it is still a leading cause of death related to skin cancer and there is a continuous elevation in its incidence.^4^ In 2010, it was reported that there were nearly 69 000 diagnoses with invasive melanoma in the USA, with about 8.7 thousand deaths from melanoma the same year.^5^ In the past, there have been no developments regarding a systemic therapeutic method with a clear clinical benefit for patients with advanced melanoma and therefore the survival rate remains poor.^6^ Hence, a comprehensive knowledge on the underlying molecular mechanisms of tumour progression is essential when finding novel paradigms for the diagnosis and therapy of melanoma.

microRNAs (miRNAs), small non‐coding RNAs of 21‐25 nucleotide‐long, influence protein expression by incompletely complementing with the 3′‐untranslated region (3′‐UTR) of target genes, and boast both oncogenic and tumor suppressive potentials in human tumors.^7^, ^8^ Multiple studies have demonstrated that miRNAs and their target genes play a vital role in a number of biological processes including cell development, proliferation, migration, invasion, apoptosis and differentiation.^9^, ^10^ A recent study has showed that miRNAs participate in malignant melanoma, which might help broaden our understanding regarding the molecular mechanisms of melanoma progression and development.^11^ The aberrant expression of microRNA‐374 (miR‐374) has been reported in many types of human tumours, including gastric cancer, lung cancer and oesophageal cancer.^12^, ^13^, ^14^ Furthermore, miR‐374 has been identified as a novel biomarker in determining the most appropriate treatment option for cancer and a novel radiation sensitizer for carbon ion beam radiotherapy.^15^ Tyrosinase (TYR) is a copper‐containing enzyme known for its participation in a variety of biological processes including wound healing, pigment production, exoskeleton fabrication and innate immunity and hardening.^16^ It has been revealed that miR‐203 regulates TYR expression and hence mediates actin‐based melanosome transport.^17^ The Wnt signalling pathway regulates normal development as well as a variety of pathologies.^18^ A previous study regarded the Wnt signalling pathway as a vital regulator of homoeostasis, which is affected in a majority of colon cancers.^19^ The association between the Wnt signalling pathway and several cell processes such as proliferation, polarity and apoptosis of cancer has been demonstrated in another previously conducted study.^20^ Based on the aforementioned findings, we suggest that both miR‐374, TYR and the Wnt signalling pathway could potentially be involved in the development of melanoma. Therefore, we conducted the present study with aims of investigating the effects of miR‐374 on proliferation, migration, invasion and apoptosis of mouse melanoma cells by mediating TYR through the Wnt signalling pathway.

## 2 MATERIALS AND METHODS

### 2.1 Ethics statement

All experimental procedures were performed on the basis of the requirements of approved by the Institutional Animal Care and Use Committee of Affiliated Hospital of Hebei Engineering University.

### 2.2 Animals

Ten healthy male nude mice weighing 20 ± 2 g and ageing 3 months were purchased from the Animal Experimental Center of Southern Medical University, 1 week prior to the experiment to adapt to the environment. The feeding environment had a humidity of 50%‐60% and a temperature of 22‐24°C with 12/12 h day/night cycle and the animals had free access to water and food.

### 2.3 Model establishment

The skin on the back portion of the mouse was sterilized with 75% ethanol and the cultured B16 cells, purchased from Shanghai Bang Jing Industrial Co., Ltd. (Shanghai, China) were extracted. The cells underwent amplification and cryopreservation in the laboratory quality control (QC) tests was conducted with a vitality of >95%. These procedures were conducted after making sure there was no bacterial, fungal and mycoplasma contamination. B16 cells were cultured in Roswell Park Memorial Institute 1640 (PRMI 1640) culture medium containing 10% foetal bovine serum (FBS), followed by routine addition of 10 U/L penicillin and 100 mg/L streptomycin. Next, the cells were cultured with 5% CO_2,_ with the number of cells adjusted to 1 × 10^5^. Subsequently, xenograft mouse models were established with the subcutaneous inoculation of 0.2 mL of cell suspension. Rate of tumour‐formation and death rate were then calculated. The mice were all tumourigenic after inoculation with no deaths reported. Afterwards, the mice were killed 3 weeks following the inoculation and the tumour mass was isolated.

### 2.4 Haematoxylin‐eosin staining

Melanoma tissues and paracancerous tissues were extracted and fixed with 3% neutral formalin, which were made into paraffin sections with a thickness of 5‐8 μm, after which haematoxylin‐eosin (HE) staining was performed. The sections were then dewaxed with xylene twice for 5 minutes each time, followed by dehydration with gradient ethanol of 100%, 95%, 80% and 75% respectively for 1 minute, after which the sections were washed with running water for 2 minutes. Next, the sections were stained with haematoxylin for 2 minutes and colour separation was conducted using 1% hydrochloric ‐ethanol followed by washing with running water for 10 seconds. Then, the sections were stained with eosin for 1 minute after which they were washed with distilled water for 1 minute. After receiving another wash with distilled water for 10 seconds, the sections were dehydrated using 95% and 100% ethanol twice for 1 minute each time. Subsequently, the sections were cleared in xylene, covered with neutral balsam, observed under a 400‐fold microscope and photographed (PH100‐2B41L‐IPL; Jiangxi Phoenix Biological Microscope Co., Ltd., Wenzhou, Zhejiang, China).

### 2.5 Immunohistochemistry

The melanoma tissues and paracancerous tissues were fixed in 10% formalin, embedded in paraffin and sliced into paraffin sections with a thickness of 4 μm. Afterwards, incubation was carried out at 60°C for 1 hour. After being dried, the sections were dewaxed with xylene three times for 10 minutes each time. Subsequently, they were dehydrated in 95%, 80% and 75% gradient ethanol respectively for 1 minute and washed with running water for 1 minute. The paraffin sections were immersed in 3% H_2_O_2 _(84885; Sigma, San Francisco, CA) and incubated at 37°C for 30 minutes, after which they were washed with PBS for 3 minutes. Subsequently, the sections were boiled with 0.01 mol/L citrate buffer at 95°C for 20 minutes and cooled down to room temperature. After being washed with PBS, the sections were blocked with normal goat serum at 37°C for 10 minutes. The sections were incubated with the primary antibody rabbit‐anti‐rat TYR (1:750; ab112, Abcam, Cambridge, MA) at 4°C overnight. After being washed with PBS, the sections were incubated with the secondary antibody goat‐anti‐rabbit (DF7852; Shanghai Yunyao Biological Technology Co., Ltd., Shanghai, China) labelled with horseradish peroxidase (HRP) at room temperature for 30 minutes. The sections were developed with diaminobenzidine (DAB) (ab64238; Abcam) and re‐stained with haematoxylin, followed by mounting. The primary antibody was then replaced by PBS as the negative control (NC), whereas the paracancerous tissues served as a positive control. Afterwards, 5‐10 visual high‐power fields were randomly selected from each section and observed under a light microscope. The cells presenting with brown stain in the nucleus were regarded as positive cells. There were no positive cells expressed as (−), positive cells ≤25% expressed as (+), positive cells of 26%‐50% expressed as (++), positive cells of 51%‐75% expressed as (+++), and positive cells >75% expressed as (++++).

### 2.6 Cell grouping and transfection

The normal cells isolated from the subcutaneous paracancerous tissues were regarded as the normal group. Meanwhile, the human melanoma cell line M21 (BeNa Culture Collection, Suzhou, Jiangsu Province, China) was selected for subsequent experiments. The B16 and M21 cells were assigned into the blank, NC, miR‐374 mimic, miR‐374 inhibitor, siRNA‐TYR and miR‐374 inhibitor + siRNA‐TYR groups (mimic: ATATAATACAACCTGCTAAGTG; inhibitor: CACTTAGCAGGTTGTATTATAT; siRNA‐TYR: TACGTCCAAGGTCGGGCAGGAAGA). Twenty‐four hours before transfection, the cells were seeded in a six‐well plate and transfected when the confluence reached 70%‐80% in accordance with the instruction of lipofectamine 2000 (11668‐019; Invitrogen, NY, CA). Two hundred and fifty microlitres of serum‐free medium Opti‐MEM (51985042; Gibco, Gaitherburg, MD) was used to dilute 100 pmol of blank, NC, miR‐374 mimic, miR‐374 inhibitor, miR‐374 inhibitor + siRNA‐TYR and siRNA‐TYR (the final concentration added to cells was 50 nmol/L), after which it was gently mixed and incubation was carried out at room temperature (about 25°C) for 5 minutes. Then, 250 µL of serum‐free medium Opti‐MEM was used for the dilution of the 5 µL of lipofectamine 2000, followed by a slight mixing and incubation at 25°C for 5 minutes. Subsequently, the two mediums mentioned above were mixed, incubated at 25°C for 20 minutes and then added into cell culture well. Following culture with 5% CO_2 _for 6‐8 hours at 37°C, the medium was replaced with a complete medium. After a 24‐48 hours of culture, the following procedures were conducted.

### 2.7 Reverse transcription quantitative polymerase chain reaction

The miRNeasy Mini Kit (217004; Qiagen Company, Hilden, Germany) was adopted to extract the total RNA from melanoma tissues and paracancerous tissues. MicroRNA‐374, TYR, β‐catenin, B‐cell leukaemia 2 (Bcl‐2), Bcl‐2 associated X protein (Bax), Low‐density lipoprotein receptor‐related protein 6 (LRP6), Leucine‐rich repeat G protein‐coupled receptor 5 (LGR5), CyclinD1 and U6 primers were designed, which were synthesized by Takara, Tykyo, Japan (Table 1). Next, the PrimeScript RT (RR036A; Takara Biotechnology Ltd., Dalian, Liaoning, China) reagent kit was adopted for the reverse transcription of the RNA into cDNA in accordance with the instruction on the kit, with a reverse transcription system of 10 µL. The reaction conditions were set as follows: reverse transcription was conducted at 37°C for 15 minutes three times and reverse transcriptase inactivation reaction was conducted at 85°C for 5 seconds. Reverse transcription quantitative polymerase chain reaction (RT‐qPCR) was then conducted with reaction liquid in accordance with the instructions of the SYBR^®^ Premix Ex Taq^TM^ II reagent kit (RR820A; Takara Biotechnology Ltd.). The reaction system was set at 20 μL including 10.0 μL of One Step SYBR^®^ RT‐PCR Buffer III, 0.4 μL of TaKaRa Ex Taq^TM^ HS, 0.4 μL of Prime Script^TM^ RT Enzyme Mix II, 0.3 μL of PCR forward primer, 0.3 μL of PCR reverse primer, 0.4 μL of ROX Reference Dye or Dye II (50×), 2 μL of total RNA and 6.2 μL of RNase Free ddH_2_O. The ABI7500 quantitative PCR instrument (7500; ABI Company, Oyster Bay, NY) was employed to conduct RT‐qPCR, with the following reaction conditions: pre‐denaturation at 95°C for 10 seconds; 40 cycles of denaturation at 95°C for 5 seconds, annealing and final extension at 60°C for 26 seconds. U6 was regarded as the internal reference of the relative miR‐374 expression and glyceraldehyde‐3‐phosphate dehydrogenase was used as the internal reference for the relative expression of TYR, β‐catenin, Bcl‐2, Bax, LRP6, LGR5 and CyclinD1. The 2^−ΔΔC^ method 21 was adopted to calculate the relative transcription level of the target gene using the following formula: △△Ct = △Ct_the experimental group_ − △Ct_the control group_ and △Ct = Ct_(target gene)_ − Ct_(internal reference)_.

**Table 1:** The primers for RT‐qPCR

Gene	Primer sequences
miR‐374	Forward: 5′‐TCCTACTCGGGTGGATATAATACAA‐3′
	Reverse: 5′‐CGAGAGCCATAACCTCGGAC‐3′
TYR	Forward: 5′‐GATGGAACACCTGAGGGACCACTAT‐3′
	Reverse: 5′‐GCTGAAATTGGCAGTTCTATCCATT‐3′
β‐catenin	Forward: 5′‐GTCAGCTCGTGTCCTGTGAA‐3′
	Reverse: 5′‐GATCTGCATGCCCTCATCTA‐3′
Bcl‐2	Forward: 5′‐TGGGATGCCTTTGTGGAACTAT‐3′
	Reverse: 5′‐AGAGACAGCCAGGAGAAATCAAAC‐3′
Bax	Forward: 5′‐CTGAGCTGACCTTGGAGC‐3′
	Reverse: 5′‐GACTCCAGCCACAAAGATG‐3′
LRP6	Forward: 5′‐AGA TCC ATC AAG TGG GTT CAT GTA‐3′
	Reverse: 5′‐AAG CGA CTT GAG CCA TCC AT‐3′
CyclinD1	Forward: 5′‐GCACGCTCGAGTGTTGAAGGGAGGTGGCAAGAG‐3′
	Reverse: 5′‐GCATTGCGGCCGCAGGATGGTTGAGGTAAGCGTGA‐3′
LGR5	Forward: 5′‐TTCACACACCCATCTCTGGT‐3′
	Reverse: 5′‐CCGGAAACAAGACACAGCTA‐3′
U6	Forward: 5′‐TCACTTGCAGGAATCGACTG‐3′
	Reverse: 5′‐ATTTGCGTGTCATCCTTGC‐3′
GAPDH	Forward: 5′‐TGCACCACCAACTGCTTAG‐3′
	Reverse: 5′‐TATGCACTGACATCTAAGTTCTTTAGCA‐3′

Abbreviations: Bax, Bcl‐2 associated X protein; Bcl‐2, B cell leukaemia 2; GAPDH, glyceraldehyde‐3‐phosphate dehydrogenase; LGR5, Leucine‐rich repeat G protein‐coupled receptor 5; LRP6, Low‐density lipoprotein receptor‐related protein 6; miR‐374, microRNA‐374; RT‐qPCR, reverse transcription quantitative polymerase chain reaction; TYR, tyrosinase.

### 2.8 Western blot analysis

The total protein extraction rapid immunofilter paper assay (RIPA) reagent kit (R0010; Beyotime Biotechnology Co., Shanghai, China) was used for the extraction of the total protein of fresh tissues and cells. The bicinchoninic acid (BCA) assay kit (P0011; Beyotime Biotechnology Ltd.) was used to determine the protein concentration. The proteins were quantified according to different concentrations. After separation of proteins by polyacrylamide gel electrophoresis, the proteins were transferred to the nitrocellulose membrane using the wet transfer method. The proteins were blocked with 5% bovine serum albumin (BSA) (Shanghai Yu Bo Biotechnology Co., Ltd. Shanghai, China) for 1 hour at room temperature. Subsequently, the proteins were probed with the diluted primary antibody rabbit‐anti‐mouse monoclonal antibody TYR (1:200, ab112), β‐catenin (1:4000, ab6302), Bcl‐2 (1:500‐1:1000, ab59348), Bax (1:1000, ab199677), LRP6 (4 µg/mL, ab51910), LGR5 (1:1000‐1:2000, ab75732) and CyclinD1 (1:1000‐1:10000, ab137875), all of which were purchased from Abcam at 4°C overnight. The membranes were washed with PBS (Shanghai Yihe Biological Technology Co., Ltd., Shanghai, China) three times, 5 minutes per time, followed by incubation with secondary antibody of goat‐anti‐rabbit IgG (1:5000; Beijing Zhongshan Biotechnology Co., Ltd., Beijing, China) labelled with HRP (HRP coupling Kit; Abcam). The membrane was immersed in enhanced chemiluminescence (ECL) solution (WBKLS0500; Pierce, Rockford, IL) for lighting, after which the images of the gels were captured in a dark room. Finally, the western blotting bands semi‐quantitative method was performed in order to measure the protein expression using the following formula: protein expression = the grey value of the target protein band/the grey value of the internal reference protein band. The measurement data were analysed using Image j software.

### 2.9 Dual luciferase reporter gene assay

microRNA.org, the biological prediction website, was applied to identify whether TYR was a direct target of miR‐374. The target sequence and mutant (MUT) sequence were designed on the basis of the binding sequences of 3′‐UTR of TYR mRNA and miR‐374. The target sequence was chemically synthesized and the restriction sites of Xho I and Not I were added at both ends of the sequence at the time of synthesis. The synthetic fragments were cloned to the PUC57 vector. After identification of positive clones and recombinant plasmid using DNA sequencing, synthetic fragments were sub‐cloned to psiCHECK‐2 vector and transformed to Escherichia coli DH5α cells to amplify plasmid. The plasmid was then extracted in accordance with the instructions mentioned on the Omega plasmid extraction kit (Shanghai Crystal Minerals Biological Technology Co., Ltd., Shanghai, China). The B26 cells were seeded in a six‐well plate with 2 × 10^5 ^per well. Following cell adherence to the well, transfection was carried out according to the aforementioned method. Once the cells were successfully transfected, the cells were cultured for 48 hours and collected. The luciferase activity of TYR 3′UTR affected by miR‐374 was detected using a luciferase assay kit (Genecopoeia, Rockville, MD). The Glomax20/20 luminometer fluorescence detector (Promega Corp., Madison, WI) was utilized to detect fluorescence intensity. Each experiment was repeated three times.

### 2.10 Cell counting kit‐8 assay

After a 48‐hour transfection, the cells were collected for cell counting. Cells were seeded in a 96‐well plate with 3 × 10^3^‐6 × 10^3^ cells per well, 0.1 mL volume per well and repeated for six wells. The cells were incubated with three time‐points set: 24, 48 and 72 hours. Next, the experiments were conducted at these three time‐points accordingly: 20 μL of 5 mg/mL cell counting kit‐8 (CCK‐8) solution were added into each well and incubation was carried out at 37°C for 4 hours. Once the culture supernatant was removed from the wells, 150 μL of dimethylsulphoxide (DMSO) was added per well. The optical density (OD) value of each well at a wavelength of 450 nm was detected in an enzyme linked immuno analyzer (NYW‐96M; Beijing Nuoyawei Instrument & Meter Co., Ltd., Beijing, China). Each experiment was repeated three times. The cell viability curve was drawn with time‐points as the abscissa and the OD value as the ordinate.

### 2.11 Scratch test

After transfection for 48 hours, the cells were seeded in a six‐well plate. After cell adherence, the medium was replaced by minimum essential medium (MEM), of which the serum concentration was 10%. When the cell confluence reached 90%‐100%, 10 μL of gunpoint was used to scratch vertically and slowly the bottom of the six‐well plate, with about 4‐5 scratches per well for the same width of each scratch. The cells were rinsed with PBS three times to wash away the drawn cells and then cultured in a cell incubator. The migration distance of cell scratch area was observed using an inverted microscope at 0 and 24 hours after scratching, with five visual fields selected, after which the images were obtained. Each group was set three wells and the experiment was repeated three times.

### 2.12 Transwell assay

After 48 hours, the cells were starved in a serum‐free medium for 24 hours, followed by digestion. After receiving two PBS washes, the cells were re‐suspended in MEM containing 10 g/L BSA (31985008; Nanjing SenBeiJia Biological Technology Co., Ltd., Jiangsu, China) with the cell density adjusted to 3 × 10^4^ cells/mL. The transwell chamber was inoculated in a 24‐well plate. The apical chamber surface of the bottom membrane of the transwell was coated with matrigel (40111ES08; Shanghai Yeasen Biotechnology Co., Ltd, Shanghai, China) diluent at 1:8 dilutions and they were dried at room temperature. Following digestion of the cells in the normal, blank, NC, miR‐374 mimic, miR‐374 inhibitor, miR‐374 inhibitor + siRNA‐TYR and miR‐374 mimic + siRNA‐TYR groups, they were washed with PBS twice. The cells were re‐suspended in MEM to adjust the cell density to 1 × 10^5^ cells/mL. Two hundred microlitres of cell suspension was added into the apical chamber of transwell which was covered with matrigel. Then 600 μL of MEM containing 20% FBS was added to the basolateral chamber of transwell. After conventional culture for 24 hours, the transwell chamber was taken out and the cells in the apical chamber were removed with the use of cotton buds. Afterwards, the cells were fixed with 4% paraformaldehyde for 15 minutes, stained with 0.5% crystal violet for 15 minutes and washed with PBS three times. Five visual fields were selected and photographed under an inverted microscope (XDS‐800D; Shanghai Cai Kang Optical Instrument Co., Ltd., Shanghai, China) to calculate the cell numbers migrating through the membranes. Each group was set three wells, the experiment was repeated three times and the mean value was obtained.

### 2.13 Flow cytometry

After transfection for 48 hours, the cells were collected and washed with cold PBS three times, followed by centrifugation, after which the supernatant was discarded. The cells were then re‐suspended with PBS and the cell density was adjusted to about 1 × 10^5^ cells/mL, with 1 mL of 75% ethanol pre‐cooled at −20°C to fix the cells at 4°C for 1 hour. Then, the ice cold ethanol was discarded following centrifugation. Then, the cells were washed with PBS twice and the supernatant was discarded. Subsequently, cells were incubated with 100 μL of RNase in a water bath at 37°C for 30 minutes under conditions void of light. To this, 400 μL of propidium iodide (PI) (Sigma, Santa Clara, CA) was added for staining. After a further incubation period devoid of light at 4°C for 30 minutes, red fluorescence was used to detect the cell cycle at an excitation wavelength of 488 nm recorded by flow cytometry. The experiment was repeated three times and the mean value was calculated.

After a 48‐hour transfection period, the cells were digested using trypsin without ethylenediaminetetraacetic acid (EDTA) and collected in the flow tube. After centrifugation, the supernatant was discarded. Cells were washed with cold PBS for three times and the supernatant was discarded after centrifugation. According to the instructions mentioned in the Annexin‐V‐fluorescein isothiocyanate (Annexin‐V‐FITC) cell apoptosis detection kit (HZB1171; Sigma, Santa Clara, CA), Annexin‐V‐FITC/PI dye liquor was prepared with Annexin‐V‐FITC, PI and hydroxyethylpiperazine‐N′‐2‐ethanesulfonic (HEPES) buffer solutions in 1:2:50. Then 100 μL of the dye liquor was used for the re‐suspension of 1 × 10^6^ cells and gently shaken for mixing. After incubation at room temperature for 15 minutes, 1 mL of HEPES buffer solution was added to cells and gently shaken for mixing. The excitation light with wavelength of 488 nm was used to excite the emission light with wavelengths of 525 and 620 nm. The scattered light and bandpass filter were employed to detect the FITC and PI fluorescence and cell apoptosis. The experiment was repeated three times and the mean value was calculated.

### 2.14 Statistical analysis

Statistical analysis was conducted using the spss 21.0 software (IBM Corp, Armonk, NY). Measurement data were presented as mean ± SD. Data differences between two groups were analysed using the *t*‐test, whereas comparisons among multiple groups were analysed using one‐way ANOVA. *P* < 0.05 was considered statistically significant.

## 3 RESULTS

### 3.1 A mouse model of melanoma was successfully established

First, the pathological characteristics of melanoma tissues and the paracancerous tissues were microscopically observed and assessed in order to confirm the successful establishment of the mouse model. Compared with the paracancerous tissues, the melanoma tissues had varying sizes and they were irregular and difficult to identify, while the presence of atypical cells was evident. There was a small number of melanin granules found in a few areas of the mice. There was large necrosis observed in the melanoma tissues and a small amount of inflammatory cell infiltration was observed in the melanoma stroma and the surrounding tissues (Figure 1). These results confirmed the successful establishment of the mouse model as evidenced by significant pathological characteristics of melanoma.

**Figure 1:** The mouse model was successfully established as evidenced by histopathological assessment in the paracancerous tissues and the melanoma tissues by haematoxylin and eosin staining (×200). HE, haematoxylin‐eosin

### 3.2 Higher positive expression rate of TYR protein was found in the melanoma tissues

Next, immunohistochemistry was conducted in order to determine whether there is a significantly different TYR expression in the melanoma tissues than that in the paracancerous tissues (Figure 2). The results revealed that the TYR positive expression was mainly detected in the cytoplasm with brown positive granules. The positive expression rate of TYR protein was (9.55 ± 1.01)% in the paracancerous tissues, which was significantly lower than that in the melanoma tissues (63.29 ± 2.48)% (*P* < 0.05). These findings suggest the important role of TYR involving the melanoma progression.

**Figure 2:** TYR is highly expressed in the melanoma tissues as shown by the immunohistochemistry results (×200). A, Immunohistochemical analysis of TYR protein in the paracancerous tissues and the melanoma tissues; B, positive expression rate of TYR protein in the paracancerous tissues and the melanoma tissues; *P < 0.05 vs the paracancerous tissues; TYR typrosinase

### 3.3 miR‐374 is poorly expressed and the Wnt signalling pathway is activated in melanoma

Reverse transcription quantitative polymerase chain reaction and western blot analysis were conducted in order to evaluate the melanoma‐induced effects through quantification of TYR, Wnt signalling pathway related factors (β‐catenin, LRP6 and LGR5), apoptosis‐related factors (Bcl‐2 and Bax) and proliferation‐related factor (CyclinD1) in the melanoma tissues and the paracancerous tissues. Compared with the paracancerous tissues, there was a significant decrease in the expression of miR‐374 and Bax in the melanoma tissues (*P* < 0.05). The expression of TYR, β‐catenin, LRP6, Bcl‐2, CyclinD1 and LGR5 increased notably, whereas the expression of Bax decreased significantly **(**all *P* < 0.05**)** (Figure 3). These results suggest that there is a poor expression of miR‐374 and the Wnt signalling pathway is activated in melanoma.

**Figure 3:** miR‐374 is poorly expressed in the melanoma tissue and the Wnt signalling pathway is activated. A, miR‐374 expression and mRNA expression of TYR, β‐catenin, LGR5, CyclinD1, LRP6, Bax and Bcl‐2 in the paracancerous tissues and the melanoma tissues measured by RT‐qPCR; B, graphs depicting GAPDH‐normalized western blot signal of TYR, β‐catenin, LGR5, CyclinD1, LRP6, Bax and Bcl‐2 in the paracancerous tissues and the melanoma tissues; C, western blot analysis of TYR, β‐catenin, LGR5, CyclinD1, LRP6, Bax and Bcl‐2 in the paracancerous tissues and the melanoma tissues; *P < 0.05 vs the paracancerous tissue; RT‐qPCR, reverse transcription quantitative polymerase chain reaction; GAPDH, glyceraldehyde‐3‐phosphate dehydrogenase; miR‐374, microRNA‐374; TYR, typrosinase; Bcl‐2, B‐Cell Leukaemia 2; Bax, Bcl‐2 associated X protein; LRP6, Low‐density lipoprotein receptor‐related protein 6; LGR5, Leucine‐rich repeat G protein‐coupled receptor 5

### 3.4 TYR is a target gene of miR‐374

Subsequently, the upstream regulatory miRNAs of TYR were explored. An online analysis software was employed and based on the findings, there was a specific binding area between TYR gene sequence and miR‐374 and TYR was verified as the target gene of miR‐374 (Figure 4A), which was further confirmed with the use of dual luciferase reporter gene assay (Figure 4B). Compared with the normal group, there was a decrease in the luciferase activity of the wild‐type (Wt)‐miR‐374/TYR in the miR‐374 mimic group (*P* < 0.05). But there was no statistical significance in luciferase activity of MUT‐miR‐374/TYR, suggesting that miR‐374 could specifically bind with the TYR gene. Based on the above findings, we concluded that TYR is a target gene of miR‐374.

**Figure 4:** miR‐374 targets TYR. A, Predict binding site of miR‐374 in TYR‐3′UTR; B, the results of luciferase activity determination; *P < 0.05 vs the normal group; miR‐374, microRNA; TYR, tyrosinase; UTR, untranslated region

### 3.5 miR‐374 negatively regulates TYR expression and inhibits the activation of the Wnt signalling pathway

Reverse transcription quantitative polymerase chain reaction and western blot analysis were conducted to further investigate that altered expression of miR‐374 can specifically induce alternation of TYR expression and the expression levels of TYR, the Wnt signalling pathway related factors (β‐catenin, LRP6 and LGR5), apoptosis‐related factors (Bcl‐2 and Bax) and proliferation‐related factor (CyclinD1) were quantified. The results (Figure 5) indicated that in comparison to the normal group, there was an evident elevation in the mRNA and protein expression of TYR, β‐catenin, LRP6, Bcl‐2, CyclinD1 and LGR5 in the remaining six groups (all *P* < 0.05), but that of Bax declined notably (all *P* < 0.05). There were no significant differences regarding the mRNA and protein expression of these genes between the blank and NC groups (*P* > 0.05). Compared with the blank and NC groups, the miR‐374 mimic and siRNA‐TYR groups showed ascended Bax expression (all *P* < 0.05) and significantly descended expression of TYR, β‐catenin, LRP6, Bcl‐2, CyclinD1 and LGR5 (all *P* < 0.05); miR‐374 expression in the miR‐374 mimic group elevated notably (*P* < 0.05), whereas there was no significant difference detected in the siRNA‐TYR group (*P* > 0.05); the expression of Bax and miR‐374 expression declined notably; and the expression of TYR, β‐catenin, LRP6, Bcl‐2, CyclinD1 and LGR5 increased significantly in the miR‐374 inhibitor group (all *P* < 0.05); miR‐374 expression in the miR‐374 inhibitor + siRNA‐TYR group decreased notably (*P* < 0.05), with no significant difference in the expression of TYR, β‐catenin, LRP6, Bax, Bcl‐2, CyclinD1 and LGR5 in the miR‐374 inhibitor + siRNA‐TYR group (all *P* > 0.05). These results suggest an indication that up‐regulation of miR‐374 can inhibit the TYR expression as well as the activation of the Wnt signalling pathway.

**Figure 5:** Restored miR‐374 inhibits TYR expression and inactivates the Wnt signalling pathway. A, miR‐374 expression and mRNA expression of TYR, β‐catenin, LGR5, CyclinD1, LRP6, Bax and Bcl‐2 of mouse cells after transfection in each group determined by RT‐qPCR; B, graphs depicting GAPDH‐normalized western blot signal of TYR, β‐catenin, LGR5, CyclinD1, LRP6, Bax and Bcl‐2 of mouse cells after transfection in each group; C, western blot analysis of TYR, β‐catenin, LGR5, CyclinD1, LRP6, Bax and Bcl‐2; D, miR‐374 expression and mRNA expression of TYR, β‐catenin, LGR5, CyclinD1, LRP6, Bax and Bcl‐2 of human melanoma cell line M2 after transfection in each group determined using RT‐qPCR; E, graphs depicting GAPDH‐normalized western blot signal of TYR, β‐catenin, LGR5, CyclinD1, LRP6, Bax and Bcl‐2 of human melanoma cell line M2 after transfection in each group; F, western blot analysis of TYR, β‐catenin, LGR5, CyclinD1, LRP6, Bax and Bcl‐2; *P < 0.05 vs the normal group; ^#^ *P* < 0.05 vs the blank and NC groups; NC, negative control; miR‐374, microRNA‐374; TYR, tyrosinane; Bcl‐2, B‐Cell Leukaemia 2; Bax, Bcl‐2 associated X protein; LRP6, Low‐density lipoprotein receptor‐related protein 6; LGR5, Leucine‐rich repeat G protein‐coupled receptor 5; GAPDH, glyceraldehyde‐3‐phosphate dehydrogenase; RT‐qPCR, reverse transcription quantitative polymerase chain reaction

### 3.6 Up‐regulation of miR‐374 and down‐regulation of TYR inhibit cell proliferation

With results identifying the aberrant expression of miR‐374 and TYR in melanoma, interests aroused considering their effects on the biological behaviours of melanoma tumour cells following delivery of miR‐374 mimic, miR‐374 inhibitor and siRNA‐TYR. Initial exploration was conducted on cell proliferation using the CCK‐8 assay. Compared with the normal group, the OD values of the cells transfected for 48 and 72 hours in the blank, NC, miR‐374 mimic, siRNA‐TYR and miR‐374 inhibitor groups were all increased (all *P* < 0.05). Compared with the blank and NC groups, the OD values of cells transfected for 48 and 72 hours in the miR‐374 inhibitor group were increased, but the OD values of cells transfected for 48 and 72 hours in the miR‐374 mimic and siRNA‐TYR groups were declined (all *P* < 0.05). There were no significant differences in the miR‐374 inhibitor + siRNA‐TYR groups compared with the blank and NC groups (*P* > 0.05) (Figure 6A). Meanwhile, the results obtained in the human melanoma cell line M21 were consistent (Figure 6B). Hence, it is elucidated that overexpression of miR‐374 and siRNA‐mediated depletion of TYR exert inhibitory effects on tumour cell proliferation in melanoma.

**Figure 6:** Overexpression of miR‐374 and siRNA‐mediated depletion of TYR suppress cell proliferation ability by CCK‐8 assay. A, Mouse cell proliferation as indicated by OD values; B, human melanoma cell line M2 proliferation as indicated by OD values; *P < 0.05 vs the normal group at 48 and 72 h; ^#^ *P* < 0.05 vs the blank and NC groups at 48 and 72 h; miR, microRNA; TYR, Tyrosinase; OD, optical value; NC, negative control; CCK‐8, Cell Counting Kit‐8

### 3.7 Up‐regulation of miR‐374 and down‐regulation of TYR suppress cell migration

Next, the scratch test was carried out in order to explore the effects of miR‐374 and TYR on tumour cell migration. The results showed (Figure 7A,B) that there was no difference in migration ability between the blank and NC groups (*P* > 0.05). Compared with the blank and NC groups, there was a significant decrease in the cell migration ability in the miR‐374 mimic and siRNA‐TYR groups, whereas the cell migration ability in the miR‐374 inhibitor group evidently decreased (all *P* < 0.05). As for cell migration ability, there was no difference in the miR‐374 inhibitor + siRNA‐TYR group, the blank and NC groups (*P* > 0.05). Similar changing tendency was observed in human melanoma cell line M21 (Figure 7C,D). These results highlight the suppressive role of miR‐374 on melanoma cell migration ability through the inhibition of the TYR expression.

**Figure 7:** miR‐374 restoration and TYR knockdown exert inhibitory effects on cell migration ability by scratch test. A, Scratch gap of mouse cells in each group under the inverted optical microscope; B, quantitative analysis of the migration rates of mouse cells; C, scratch gap of human melanoma cell line M2 in each group under the inverted optical microscope; D, quantitative analysis of the migration rates of human melanoma cell line M2; *P < 0.05 vs the blank and NC groups; miR, microRNA; TYR, Tyrosinase; NC, negative control

### 3.8 Up‐regulation of miR‐374 and down‐regulation of TYR suppress cell invasion

The tumour cell invasive ability was then evaluated using transwell assay after transfection. The results (Figure 8A,B) indicated that there was no difference in invasion ability between the blank and NC groups (*P* > 0.05). Compared with the blank and NC groups, the invasion ability in the miR‐374 mimic and siRNA‐TYR groups decreased significantly, whereas the invasion ability in the miR‐374 inhibitor group increased (all *P* < 0.05). The invasion ability of the miR‐374 inhibitor + siRNA‐TYR group showed no difference compared with the blank and NC groups (*P* > 0.05). Consistently, the human melanoma cell line M21 showed the identical tendency in migration as in invasion after treatment (Figure 8C,D). Hereby, available evidence further proves the adverse effects of up‐regulated miR‐374 and silenced TYR on melanoma cell invasion.

**Figure 8:** Cell invasion ability is weakened by overexpressed miR‐374 and silenced TYR by transwell assay. A, Invasive ability of mouse cells receiving different treatments confirmed by the transwell assay under the inverted optical microscope; B, quantitative analysis of the invasive mouse cells; C, invasive ability of human melanoma cell line M2 receiving different treatments confirmed by the transwell assay under the inverted optical microscope; D, quantitative analysis of the invasive human melanoma cell line M2; *P < 0.05 vs the blank and NC groups; miR, microRNA; TYR, Tyrosinase; NC, negative control

### 3.9 Up‐regulation of miR‐374 and down‐regulation of TYR decrease cell proportion at G0/G1 phase and increase cell proportion at S phase

Whether miR‐374 and TYR can be responsible for cell cycle distribution in melanoma was the next research focus and flow cytometry was introduced to aid this process. The results revealed (Figure 9A,B) that cell proportions at G0/G1 phase in the normal, blank, NC, miR‐374 mimic, miR‐374 inhibitor, siRNA‐TYR and miR‐374 inhibitor + siRNA‐TYR groups were (59.46 ± 6.45)%, (85.01 ± 4.42)%, (85.48 ± 4.47)%, (72.33 ± 7.33)%, (97.78 ± 1.90)%, (72.44 ± 7.43)% and (85.49 ± 2.48)% separately and cell proportions at the S stage were (37.99 ± 3.65)%, (12.53 ± 1.10)%, (12.59 ± 1.31)%, (25.01 ± 2.43)%, (0.07 ± 0.01)% and (25.21 ± 5.3)%, (12.53 ± 1.21)%. Compared with the normal group, the main change of cell cycle in the blank, NC, miR‐374 mimic, miR‐374 inhibitor, siRNA‐TYR and miR‐374 inhibitor + siRNA‐TYR groups was the extension of G0/G1 phase (increase of cell proportion) and shrinkage of S phase (decrease of cell proportion) (all *P* < 0.05). Compared with the blank and NC groups, the miR‐374 mimic and siRNA‐TYR groups presented with a shrinkage at G0/G1 phase (decrease of cell proportion) and extension of S phase (increase of cell proportion), whereas the miR‐374 inhibitor group showed extension of G0/G1 phase (increase of cell proportion) and shrinkage of S phase (decrease of cell proportion) (all *P* < 0.05). There was no difference in the miR‐374 inhibitor + siRNA‐TYR group as compared to the blank and NC groups (*P > *0.05). There was no significant difference observed in G2 stage in each group (*P > *0.05). The results with regard to the human melanoma cell line M21 were in line with the above results in mouse cell line (Figure 9C,D). These findings were indicative of the involvement of miR‐374 in melanoma cell cycle distribution by targeting TYR.

**Figure 9:** Up‐regulation of miR‐374 and silencing of TYR are responsible for promoting melanoma cell cycle arrest by flow cytometry. A, Diagram of mouse cell cycle distribution in each group; B, percentage of mouse cell cycle distribution in each group; C, diagram of cell cycle distribution of human melanoma cell line M2 in each group; D, percentage of cell cycle distribution of human melanoma cell line M2 in each group; *P < 0.05 vs the normal group; ^#^ *P* < 0.05 vs the blank and NC groups; miR, microRNA; TYR, Tyrosinase; NC, negative control

### 3.10 Up‐regulation of miR‐374 and down‐regulation of TYR promote cell apoptosis

Lastly, Annexin‐V‐FITC/PI double staining was conducted to detect the effects of miR‐374 and TYR on melanoma cell apoptosis. The results (Figure 10A,B) presented with a decrease in the cell apoptosis rate in the blank, NC, miR‐374 mimic, miR‐374 inhibitor, siRNA‐TYR and miR‐374 inhibitor + siRNA‐TYR groups in comparison with the normal group (all *P* < 0.05). When compared to the blank and NC groups, the miR‐374 inhibitor group was found to have declined cell apoptosis rate while the miR‐374 mimic and siRNA‐TYR groups showed the opposite trend (all *P* < 0.05). There was no significant difference in cell apoptosis rate in the miR‐374 inhibitor + siRNA‐TYR, blank and NC groups (*P* > 0.05). In addition, the human melanoma cell line M21 presented with similar changing tendency (Figure 10C,D). The aforementioned results demonstrate that weakened cell apoptotic ability in melanoma can be reversed by the up‐regulation of miR‐374 and silencing of TYR.

**Figure 10:** Cell apoptosis is promoted by up‐regulated miR‐374 and silenced TYR. A, Distribution of live, apoptotic and necrotic mouse cells detected using Annexin‐V‐FITC/PI double staining; B, apoptosis rate of mouse cells in each group; C, distribution of live, apoptotic and necrotic cells of human melanoma cell line M2 detected using Annexin‐V‐FITC/PI double staining; D, apoptosis rate of human melanoma cell line M2 in each group; *P < 0.05 vs the normal group; ^#^ *P* < 0.05 vs the blank and NC groups; miR, microRNA; TYR, Tyrosinase; FITC, fluorescein isothiocyante; PI, propidium iodide; NC, negative control

## 4 DISCUSSION

Melanoma is the third most common basal diagnosis in patients with cerebral metastases after breast and lung cancer.^22^ The critical role played by miRNAs in the inhibition of the malignant development of human cancer by targeting tumour suppressor genes or oncogenes has been highlighted in numerous studies over the past 10 years.^23^ Therefore, in the present study, we investigated the effects of miR‐374 on mouse melanoma cells and found that miR‐374 can inhibit proliferation, migration and invasion and promote apoptosis of mouse melanoma cells through inactivating the Wnt signalling pathway by negatively regulating TYR expression.

Initially, one of the most important results revealed that compared with the paracancerous tissues, the melanoma tissues showed higher TYR expression and lower miR‐374 expressions and that TYR is the target of miR‐374. miRNAs are involved in a broad spectrum of pathological and physiological processes, including cancer‐related functions, such as cells proliferation, cells cycle, migration, invasion, immune evasion and drug resistance.^24^ Based on previously conducted studies, higher TYRP1 expression was found in patients with primary melanomas accompanied with a significantly declined survival rate and increased TYR expression during tumourigenesis.^25^, ^26^ It has also been reported that TYR expression is significantly increased in both the photo‐exposed and the photo‐protected human skin, indicating that TYR may play a crucial role in the mediation of the ethnic differences in constitutive skin pigmentation and melanogenesis.^27^ Consistently, Dong et al provided evidence that there is a remarkable decrease in miR‐34b/c expression in uveal melanoma cells and that the up‐regulation of miR‐34b/c resulted in the suppression of cell proliferation and migration by targeting c‐Met in uveal melanoma,^28^ which further proved our conclusion, suggesting that miR‐374 could directly target TYR gene and thereby regulate cell proliferation, migration, invasion and apoptosis.

Moreover, our study also revealed that there was a decreased expression in TYR, β‐catenin, LRP6 and LGR5 in the miR‐374 mimic and siRNA‐TYR groups. β‐catenin is an integral structural component of cadherin‐based adherens junctions and the critical nuclear effector of canonical Wnt signalling in the nucleus.^29^ Low‐density lipoprotein receptor‐related protein 6 is an essential co‐receptor for the Wnt signalling pathway.^30^ Leucine‐rich repeat G protein‐coupled receptor 5 is a marker of adult stem cells that participates in carcinogenesis but also maintains stemness by activating the Wnt/β‐catenin signalling in breast cancer.^31^ Multiple researches have demonstrated the high metastasis propensity of melanoma.^32^ The Wnt signalling pathway is considered as one of the critical signalling cascades and its aberrant activation affects melanoma development.^33^ In addition, it has been demonstrated that up‐regulation of miR‐34a negatively mediates the Wnt/β‐catenin signalling pathway in liver tumourigenesis, making it a novel biomarker in cancer therapy.^34^ The down‐regulation of Wnt1, a target gene of miR‐34a, could result in the inactivation of the Wnt signalling pathway, suppressing the progression of breast cancer.^35^ Furthermore, there is a close correlation between the down‐regulation of TYR and the inhibition of melanogenesis.^36^ Based on the aforementioned findings, we came to the conclusion that β‐catenin, LRP6 and LGR5 are involved in the Wnt signalling pathway and the inactivation of which may be linked to the up‐regulation of miR‐374 and down‐regulation of TYR, eventually leading to a decrease in the expression of β‐catenin, LRP6 and LGR5 and thereby affecting the development of melanoma.

Consequently, we found that up‐regulation of miR‐374 and down‐regulation of TYR led to the inhibition of cell proliferation, migration, invasion and promoted apoptosis with increased expression of Bax and decreased Bcl‐2 and CyclinD1 expression. CyclinD1 is a crucial promoter of the cell cycle and a predictive and prognostic factor in multiple kinds of cancers.^37^ Bcl‐2 is an anti‐apoptosis protein, whose expression has the ability to directly prevent cell apoptosis by limiting the pro‐apoptosis member activity of Bcl‐2 family, whereas Bax is pro‐apoptotic factor of the Bcl‐2 family that regulates the programmed cell death.^38^, ^39^ In the same miRNA family, there is evidence showing that the loss of miR‐145, miR‐133a and miR‐133b could promote cell proliferation, migration, invasion and cell cycle progression in vitro.^40^ A study conducted by Zhen et al found that PDCD4‐induced miR‐374a‐CCND1‐pPI3K/AKT‐c‐JUN feedback loop could potentially result in the suppression of suppress growth, metastasis as well as chemotherapy resistance of nasopharyngeal carcinoma.^41^ There is also a similar study indicating that miR‐374a can promote gastric cancer cell proliferation, migration and invasion by directly targeting SRCIN1.^42^ All of these findings provided a possible interpretation for our conclusion.

In conclusion, this study provided evidence that up‐regulated miR‐374 can inhibit in vitro proliferation, migration, invasion and promote apoptosis of mouse melanoma cells by targeting TYR gene via the Wnt signalling pathway, suggesting that miR‐374 could be a new potential biomarker in the diagnosis and treatment of melanoma. However, whether miR‐374 has the ability to mediate other genes related to mouse melanoma cell proliferation and apoptosis via the Wnt signalling pathway remains unclear. Therefore, further studies are required to rule out the influence of other target genes of miR‐374 and to clarify the specific mechanisms on how miR‐374 regulates cell proliferation and apoptosis of melanoma.

## CONFLICT OF INTEREST

The authors have declared that no competing interests exist.

## AUTHOR CONTRIBUTION

X‐JL, Z‐FL and Y‐YX designed the study, ZH and Z‐JL collated the data, designed and developed the database. Z‐FL and ZH carried out data analyses. X‐JL and Y‐YX conceived and designed the experiments. All authors read and approved the final manuscript.
